The article "The Utilization Ratio and Interoperability of Corporate-Level XBRL Classification Standard Elements in China" was published in 2022. Journal: Comput Intell Neurosci.

# The Utilization Ratio and Interoperability of Corporate-Level XBRL Classification Standard Elements in China

**DOI:** 10.1155/2022/4897908

**Published:** 2022-10-06

**Authors:** Xin Song, Zijie Ding, Chao Liu, Qiongyao Zhang

**Affiliations:** ^1^Business School, University of Shanghai for Science and Technology, Shanghai 200093, China; ^2^School of Accounting, Nanjing University of Finance & Economics, Nanjing 210000, China; ^3^Department of Accounting and Taxation, Robert Morris University, Moon Township, PA 15108, USA

## Abstract

Given the rapid development of the digital industry, the international use of XBRL as a computer language for the exchange of corporate financial data is of great significance in promoting the standardization of financial data. This paper provides an in-depth study and quantitative measurement of the applicability of the Chinese XBRL common taxonomy elements in enterprises, examining the interoperability of the elements between enterprises and the possible absence and ambiguity of the elements. The research study shows significant differences between the elements of XBRL defined in the general classification standard and the elements used in financial reports of listed companies in China. Furthermore, the quantitative interoperability model results show significant differences in the interoperability of elements between companies in the same industry and the same category of industries. Therefore, updates to the Chinese XBRL taxonomy should start from the underlying logic of accounting and improve the process of calling the elements in the accounting process.

## 1. Introduction

Extensible business reporting language (XBRL) is an internet-based, cross-platform computer language for preparing, disclosing, and using financial reports. The adoption of XBRL in China has been propelled by significant policy initiatives of the Chinese government, notably the 2015 edition of Generic Classification Standard for Enterprise Accounting Standards in April 2015, the 13th Five-Year Plan for Accounting Reform and Development in October 2016, and the outline of the 14th Five-Year Plan for Accounting Reform and Development in November 2021, all issued by the Chinese Ministry of Finance [1]. These government policies highlight the importance of XBRL-based reporting for the future development of financial reporting and the standardization of corporate accounting data in China.

XBRL has been vigorously promoted by Chinese national policies to harvest its potential benefits of presenting high-quality accounting information, providing real-time monitoring of management, and continuous auditing of enterprises (Alison and Mike [2]; Bernhard and Thomas [3]; Jacqueline et al. [4]; Liu and Xue [5]; Matteo and Diego [6]; Zhang [7]; Zhang and Ye [8]). XBRL reporting requires interactive data tagging of financial statements, which allows investors to extract information and compare and analyze different companies and periods more efficiently. XBRL reporting can therefore improve the accessibility and usefulness of data in financial statements, encouraging investors to search for company-level fundamentals and conduct in-depth analysis (Zhang et al. [9]). The effectiveness and standardization of financial statement information disclosure are crucial for the decision usefulness of information (He et al., 2015 [10]). Efficient and transparent information disclosure can reduce the information asymmetry between companies and stakeholders (Liu, 2013 [11]; Theresa Dunne, 2013 [12]).

However, XBRL has certain shortcomings and deficiencies in both technology and application (Mao and Zhang [13]; Purnendu et al. [14]), such as the issues of insufficient XBRL elements and element redundancy (Gao and Zhang [15]). The overuse of customized elements deteriorates investors' understanding of a company's financial position and performance, making it more difficult to curb management's hoarding of bad news. The results could lead to increased levels of investor perception of future collapse risk (Roman et al. [16]). The XBRL extensibility feature allows companies to customize the taxonomy to meet their unique reporting requirements. The elements defined by the taxonomy cannot be standardized across industries (Li and Yi [17]). Still, differences between multiple XBRL taxonomies and instance documents make it difficult to compare documents (Roger et al. [18], Chowdhuri et al. [19]), which compromises the interoperability of XBRL data and the relevance of financial reporting (Pei and Vasarhelyi [20]).

Most of the existing literature on XBRL interoperability surveys a sample of items disclosed in the annual reports of listed companies, manually comparing with the elements defined in the standard. In this paper, we take a modeling approach to construct a quantitative analysis model of XBRL interoperability. The disclosure items of all listed companies in China are included in the scope of the study. The quantitative analysis is carried out using an elemental interoperability model, modeling XBRL elements defined in the standard.

This study documents the insufficiency and redundancy of XBRL elements used in China. We examined the commonality of the elements within and between industries and evaluated the standardization of elements. We made suggestions regarding how to adjust the elements of the XBRL taxonomy to improve the interoperability of financial reporting elements and the accuracy of element compilation in XBRL software.

This study contributes to the XBRL and information systems literature twofold. First, it proposes and tests an interoperability model for analyzing XBRL elements. Second, it examines data from all listed companies in China (for one year), alleviating possible sampling biases in previous studies.

## 2. XBRL Data Structure and the Modeling Approach

### 2.1. Components of XBRL

XBRL consists of three parts: XBRL technical specifications, XBRL taxonomies, and XBRL instance documents. The XBRL technical specification is the core and foundation of XBRL, defining the coding and usage rules for the other two parts of XBRL and regulating the various elements and attributes that express the information. The taxonomy is a concrete description of the technical specification, consisting of a schema document and a link library, where the schema document defines the concept of financial reporting elements and extended link roles, and the link library defines the links between the elements. The XBRL instance document is a concrete representation of the financial statements created by the reporting company [21].

### 2.2. The Data Structure of XBRL

Information data can be divided into three categories according to the storage form: structured data, unstructured data, and semistructured data. Semistructured data, as defined by Abiteboul [22], are in-between structured data with a fixed schema and unstructured data with no schema at all. The dual properties of semistructured data offer flexibility for complex distributed information environments. Semistructured data are suitable for multidimensional information. XBRL data fall into the category of semistructured data. These advantages make XBRL applications attract much attention, and the composition of its data is also directly related to XBRL. The way the taxonomy is modeled is relevant.

The technical core of XBRL is XML, a technology that allows data to be identified and categorized in a unified way so that it can be quickly read by the corresponding software, enabling data to be entered and reused once. The current XML (extensible markup language) document object model (DOM) is a representation model that combines trees and objects in a way that is suitable for storing semistructured data. XML is a meta-annotation language that permeates unstructured data with structure, highlighting the relationships between data. It provides a unified way to describe and exchange application-independent structured data, simplifies data representation and interaction, allows for more accurate declarations of content, and facilitates the cross-platform search for more valuable results.

### 2.3. The Dimensional Modeling Approach of XBRL

Both the financial reporting taxonomy framework (FRTA) and the Chinese taxonomy prohibit the use of tuples in multidimensional model data, so the XBRL specification introduces XBRL dimensions to address the complex concept of multidimensionality. The optional functional module XBRL dimensions put additional information into the contextual elements so that programs can read the data and obtain the meaning and contextual significance of the elements. The concept of dimensional modeling was developed during the development of the construction of data warehouses, where data warehouses or data marts are built based on tables of facts and dimensions (Chen [23]). There are three ways of modeling multidimensional information: the data item approach, the tuple approach, and the dimensional approach. Dimensional modeling techniques are used in the XBRL generic taxonomy to construct multidimensional tables, i.e., to specify dimensions. The dimensions used in the generic taxonomy are divided into generic and nongeneric dimensions in terms of their scope of application: generic dimensions can be applied by the reporting company to any essential item as required, for example, “dimensions—retrospective application and retrospective restatement,” nongeneric dimensions are mainly used to describe specific report items, for example, “dimension—supplier category.”

### 2.4. XBRL Common Taxonomy Modeling Approach

When mapping taxonomies, the modeling methods for the common taxonomies are considered. The generic taxonomies are organized per the presentation requirements of China's enterprise accounting standards and are structured into element and extended link roles. Depending on the object, the generic taxonomies modeling methods are divided into three categories: (1) modeling of the main financial statements (excluding notes), (2) modeling of notes using dimensions, and (3) modeling of general notes. The first and third modeling approaches are simple two-dimensional, with a sample element in the table header plus a core currency-type element. The second modeling approach, using dimensional note modeling, has a complex modeling approach with multiple mappings, including multiple data types, namely data descriptions in multiple dimensions, plus a description object as a currency-type element. As seen from the three modeling approaches, the study of elements for generic taxonomies is primarily a study of monetary-type elements. In contrast, dimensional elements such as abstract elements are nondisclosed objects for axial elements.

## 3. XBRL Element Interoperability Research Methodology

### 3.1. Sample Selection and Data Sources

The China Securities Regulatory Commission (CSRC) industry classification guidelines divide all listed companies in China into 19 industrial categories: *A*, agriculture, forestry, animal husbandry, and fishery; *B*, mining; *C*, manufacturing; *D*, electricity, heat, gas, and water production and supply; *E*, construction; *F*, wholesale and retail; *G*, transportation, storage, and postal services; *H*, accommodation and catering; I, information transmission, software, and information technology services; *J*, finance; *K*, real estate; *L*, leasing and business services; *M*, scientific research and technical services; *N*, water, environment, and public facilities management; *O*, residential services, repairs, and other services; *P*, education; *Q*, health and social work; *R*, culture, sports, and recreation; *S*, general. A total of 16 industries were selected for the study, and 3,699 sample companies were chosen by excluding the financial sector, residential services, the general category, companies listed on the Science and Technology Innovation Board, B-share companies, and Special Treatment (ST) companies. The 2020 annual reports issued by these 3,699 companies in 2021 were studied for this study.

This paper focuses on XBRL elements. The general classification criteria should be designed to apply to all companies in all industries, making the financial reporting elements comparable. Therefore, we selected all the companies from the selected industries.

## 4. Research Methodology

### 4.1. Methodology for the Selection of XBRL Common Taxonomy Elements

XBRL processes semistructured data and is not limited to a two-dimensional data structure, allowing for the linking of multidimensional data. This data model allows for different tags and definitions in the composition of the XBRL taxonomy elements. The elements of the generic taxonomy in Table 1 are classified and filtered, and those elements in the XBRL generic taxonomy definition format with an element type of monetary-type *X* are selected for the study. We focus on monetary elements because the abstract elements and other dimensional elements are not disclosure objects.

We started with 2045 elements of the common currency type and excluded 1820 elements from the notes to the financial statements. A total of 225 elements of the currency type of the consolidated financial statements were selected. The total number of financial statement elements disclosed by listed companies is 295.

## 5. Methodology for Matching XBRL Elements in Financial Reports of Listed Companies

The XBRL consolidated statement core elements we selected in the previous step are matched one-to-one with the financial statement elements disclosed by the listed company. If the match is successful, a score of 1 is assigned to the element. Suppose an element does not meet the definition criteria for a currency-based element. In that case, it can be considered as an element that exceeds the XBRL classification criteria, and the item is treated as an extended element. Only currency-type elements are matched in this paper, not axis elements.

### 5.1. Metric Model Proposal and Definition of Metrics

Models 1–4 measure the interoperability of XBRL with financial statements–the extent to which the XBRL instance document elements can cover real financial statements, reflecting the quality of the XBRL taxonomy element definitions. Let = {|be a financial statement, and *i* = 1 to *n*} be a set of financial statements. Let || represent the number of generic taxonomy elements used in ||. || represents the number of custom elements for a company and defines || as || + ||. Interoperability between the statements is based on shared data elements.

Two statements *d*_*i*_ and *d*_*j*_and their interoperability *I*_*i*,*j*_ can be defined as

(1) $$\begin{array}{c} I_{i,j}=\frac{\left|d_{i}\cap d_{j}\right|}{\sqrt{\left|d_{i}\right|\left|d_{j}\right|}}\text{.} \end{array}$$

Interoperability of the elements of the XBRL common taxonomy for financial reporting *I*_*i*,*j*_′ can be defined as

(2) $$\begin{array}{c} I_{i,j}^{\prime }=\frac{\left|d_{i}^{g}\cap d_{j}^{g}\right|}{\sqrt{\left|d_{i}^{g}\right|\left|d_{j}^{g}\right|}}\text{.} \end{array}$$

Two-pair interoperability is defined as the average pairwise interoperability of all pairs. Interoperability is essential when investors and analysts compare the financial statements of two companies. When analyzing the financial statements of *K* companies at the same time, the interoperability of K companies can be defined as

(3) $$\begin{array}{c} I_{i_{1}\ldots \ldots i_{k}}=\frac{\left|d_{i_{1}}\cap \ldots \ldots \cap d_{i_{k}}\right|}{\sqrt{\left|d_{i_{1}}\right|\ldots \ldots \left|d_{i_{k}}\right|}}\text{.} \end{array}$$

Then, the interoperability of the elements of the XBRL common taxonomy for financial reporting of *K* companies can be defined as

(4) $$\begin{array}{c} I_{i_{1}\ldots \ldots i_{k}}^{\prime }=\frac{\left|d_{i_{1}}^{g}\cap \ldots \ldots \cap d_{i_{k}}^{g}\right|}{\sqrt{\left|d_{i_{1}}^{g}\right|\ldots \ldots \left|d_{i_{k}}^{g}\right|}}\text{.} \end{array}$$

The interoperability of *K* companies can be defined as the average of the interoperability between all *K* tuples.

## 6. Results of the XBRL Element Utilization and Element Interoperability Study

### 6.1. XBRL Element Utilization Study Results

We found elements that are not disclosed by enterprises as defined in the XBRL generic taxonomy were identified in both financial statement elements and note elements, such as “assets classified as held for sale,” “long-term employee compensation payable,” and “amounts at fair value through profit or loss,” “net of tax of other comprehensive income attributable to minority shareholders” in the consolidated statements of operations, “amounts at fair value through profit or loss,” “amounts after tax of other comprehensive income attributable to minority shareholders,” and “amounts at fair value through profit or loss,” “amount at fair value through profit or loss,” “other comprehensive income attributable to minority shareholders, net of tax,” and “effect of business combinations under common control.” These elements are all parts of the generic classification but are not used by companies in the disclosure process. Also, during the matching and statistical process, we found that companies disclosed elements are not defined in the XBRL generic taxonomy, such as “precious metals,” “subrogation receivables,” and “pledged loans to policyholders” in the balance sheet.

All of the above matched and counted elements of the XBRL financial statement common taxonomy were analyzed for usage and utilization (as shown in Figures 1 and 2). The graph of element usage corresponds to the “sum” item of the element statistics in the descriptive analysis, as seen in Figure 1. There are 60–70 high-frequency elements and 20–30 medium-frequency elements. These high-frequency elements account for approximately 44.44% of the elements in the general classification. The 70 or so elements on the far right-hand side of the horizontal axis are used quite infrequently, with ten elements having a usage rate close to 0. The proportion of low-frequency elements is approximately 35.56%, and approximately 18.67% of the generic elements cannot be matched to the elements of the corporate consolidated statement.

The interpretation of this graph provides further evidence of the high utilization of some elements of the XBRL generic taxonomy and the low utilization of most elements of the XBRL generic taxonomy.

## 7. Results of the XBRL Common Taxonomy Element Interoperability Study

### 7.1. Results of the Study on Interoperability of Elements within the Industry

According to the interoperability model, all elements of the financial report disclosures were processed. The MATLAB software package was used for round-robin processing to eliminate companies whose conditions did not match. We analyzed a total of 1,402 companies. Of these, 40 were in industry A, 71 in industry B, 2,436 in industry C (only 150 companies were randomly selected to reduce the sample size), 115 in industry *D*, 96 in industry *E*, 162 in industry F, 103 in industry *G*, 7 in industry H, 292 in industry I, 108 in industry K, 52 in industry *L*, 58 in industry *M*, 69 in industry N, 11 in industry P industry, 10 in industry *Q*, and 58 in industry R. In each of these 16 industries, companies in each industry are compared on a two-by-two element basis to find the interoperability value between the two companies. There are interoperability indicators for each industry. (*n* = number of listed companies in each industry).

Figures 3–6 show the variation in interoperability within industries, with interoperability values ranging from 0.25–0.35 for the F industry, 0.35–0.4 for the K industry, and 0.32–0.36 for the C industry. Industry K has the most significant fluctuations in elemental interoperability among the 16 industries, with a range of approximately 0.28. And the interoperability of the *Q* industry is the least volatile, with a range of approximately 0.1. The comparison chart clearly reflects the differences in the interoperability of XBRL elements disclosed by companies in the same industry and in different industries.

### 7.2. Results of Interindustry Element Interoperability Studies

When further investigating the interoperability of XBRL elements across different industries, we randomly picked one company from different industries for a total of 16 companies and then performed a two-by-two interoperability valuation to obtain a total of = 120 values of interindustry interoperability. As seen in Figure 7, the first 16 sets of data are the mean interindustry interoperability values, and the last column is the mean of the 16 interindustry interoperability values, which is significantly smaller. This suggests that there are industry-level differences in XBRL interoperability. The interindustry variance of listed companies' interoperability was calculated to verify the interindustry fluctuations in XBRL element interoperability (see Figure 8). Figures 8 and 9 show large fluctuations in the variance of interoperability between industries, further validating the existence of industry-level differences in the interoperability of XBRL elements.

We used Matlab to perform round-Robin counting to find and compare values by increasing the number of companies as a robustness test while examining the results of interoperability of XBRL elements at the financial statement level. First, the first two companies were selected to find the interoperability of any seven companies from each of the 16 industries. Then, a third company was added to find the interoperability until 112 companies were added. The interoperability is shown in Figure 10. The interoperability of the first two companies at the financial statement level is close to 0.5. As the number of companies increases, the interoperability between companies gradually decreases, and after all 112 companies are added, this interoperability decreases to below 0.2. The more companies are compared on an elemental basis, the less comparable they become. The interoperability of XBRL elements at the financial statement level is lower across industries than for the same industry.

## 8. Research Findings and Implications

This paper examines the matching of the XBRL elements in China's newly promulgated Common Criteria for Enterprise Accounting Standards with the items disclosed in the financial statements of listed companies. In the process of matching, we found that the elements of the generic standard defined in XBRL differ excessively from those disclosed in the financial statements of listed companies. A possible reason is that they are defined in two completely different directions. For example, in the Note_Inventory element, companies disclose along the line of “in-process,” “inventory,” and “raw materials.” At the same time, the classification standard uses elements such as “opening balance of inventories,” “current increase in inventories,” and “current decrease in inventories.” This challenges the applicability of the elements defined in the common taxonomy to the enterprise.

Our quantitative analysis of XBRL element usage shows that the XBRL common taxonomy elements contain elements that are not used by companies that account for approximately 19% of the total common taxonomy elements, suggesting redundancy of elements. At the same time, companies also disclose elements not defined in the XBRL taxonomy, suggesting there is a shortage of elements. Elements with a utilization rate of over 50% represent approximately 44% of the GCS elements, while around 35% of the elements are underutilized, and the rest are missing in corporate financial statements.

This paper examines the interoperability of elements, redundant, and missing elements. The study finds that the interoperability of listed companies' disclosure elements fluctuates around 0.19 between enterprises in the same industry. The interoperability of elements at the interindustry level fluctuates more, at around 0.33, indicating that the interoperability of XBRL elements for financial reporting within industries is higher than interindustry interoperability. The matching rate between XBRL elements and financial statement elements is low. And there are problems such as incomplete, untimely, and insufficiently relevant disclosure of financial statement information, which leads to a decline in the comparability of data disclosed in an enterprise's XBRL financial report, and the quality of financial statement disclosure, and users of financial statements. The information obtained by financial statement users is messy, exacerbating the information asymmetry between enterprises and external stakeholders.

The XBRL taxonomy should be revised to improve the disclosure of financial statements of listed companies by making timely deletions and additions in line with adjustments to accounting standards. The XBRL taxonomy should be revised following the adjustment of accounting standards. The solution to the financial statement level should be addressed from the underlying accounting logic, i.e., the element definition should stem from the financial statement level to the accounts level. Accounting and finance professionals should take additional training to understand the elements. In the era of big data, the road to data standardization is inevitable. The standardization and improvement of XBRL standards can promote the better development of accounting information systems. Regulators should further improve and develop more comprehensive and applicable XBRL element standards to improve the transparency of market information, create a good market environment, and facilitate effective communication between companies and stakeholders.

## Figures and Tables

**Figure 1:** XBRL common taxonomy element usage.

**Figure 2:** XBRL common taxonomy element utilization rate.

**Figure 3:** Interoperability results for listed companies in K E D B industries.

**Figure 4:** Interoperability results for companies listed in the N R F Q industries.

**Figure 5:** Interoperability results for companies listed in the M G P A industries.

**Figure 6:** Interoperability results for listed companies in the C H I L industries.

**Figure 7:** Comparison of mean values of interoperability of listed companies between industries.

**Figure 8:** Comparison of interoperability variance of listed companies between industries.

**Figure 9:** Comparison of mean and variance of interoperability of listed companies between industries.

**Figure 10:** Elemental interoperability results at the financial statement level.

**Table 1:** Definitions of XBRL common taxonomy elements.

Element type	Meaning	Element type	Meaning
Text block	Text blocks, which can contain tables inside	Shares	Number of shares
Text	Text, internal plain text	table	Dimensionalised tables
yyyy-mm-dd	Point in time	Axis	Axes of the dimensionalisation table
X	Monetary	Member	Members on the dimensionalisation table axis
X.XX	Numerical	Lineitems	Presentation matters in dimensionalised tables

## Data Availability

The dataset can be accessed upon request.
